This article has been retracted.

# Neonicotinoid’s resistance monitoring, diagnostic mechanisms and cytochrome P450 expression in green peach aphid [*Myzus persicae* (Sulzer) (Hemiptera: Aphididae)]

**DOI:** 10.1371/journal.pone.0261090

**Published:** 2022-01-12

**Authors:** Muhammad Umair Sial, Khalid Mehmood, Shafqat Saeed, Mureed Husain, Khawaja Ghulam Rasool, Abdulrahman Saad Aldawood

**Affiliations:** 1 Institute of Plant Protection, Muhammad Nawaz Shareef (MNS) University of Agriculture Multan, Punjab, Pakistan; 2 Key Laboratory of Control of Biological Hazard Factors (Plant Origin) for Agriproduct Quality and Safety, Ministry of Agriculture and Rural Affairs of the People’s Republic of China, Institute of Plant Protection, Chinese Academy of Agricultural Sciences, Beijing, PR China; 3 Plant Protection Department, College of Food and Agriculture Sciences, King Saud University, Riyadh, Saudi Arabia; King Khalid University, SAUDI ARABIA

## Abstract

Green peach aphid [*Myzus persicae* (Sulzer) (Hemiptera: Aphididae)] is a significant pest with a known history of insecticide resistance. Neonicotinoids could manage this pest; however, their frequent use led to the evolution of resistance in field populations of *M*. *persicae*. Toxicity data for neonicotinoid insecticides synergized with pipernyl butoxide (PBO) in a field population (FP) were collected and compared to a laboratory susceptible clone (SC) of aphids. The enhanced expression of metabolic resistance-related cytochrome P450 gene *CYP6CY3* and an arginine-threonine substitution were detected in FP, causing a single point mutation (R81T) at *β1* subunit of nicotinic acetylcholine receptor (nAChR) within D loop. High level of resistance to imidacloprid was developed in FP with 101-fold resistance ratio and moderate resistance level (10.9-fold) to acetamiprid. The results of PBO synergized bioassay suggested that cytochrome P450 enzymes were involved in the resistance to neonicotinoids. The mRNA transcriptional level of *CYP6CY3* gene was significantly higher (3.74 fold) in FP compared to SC. The R81T mutation associated with neonicotinoid resistance had 26% resistant allele frequency in FP. Both P450 enzymes and R81T mutation of nAChR were found in field-evolved neonicotinoid resistance. It is concluded that field-evolved resistance in green peach aphid could be managed by using appropriate synergists such as PBO.

## Introduction

Green peach aphid [*Myzus persicae* (Sulzer) (Hemiptera: Aphididae)] is a serious pest of different crops globally [1]. It damages >400 plant species in 40 families and transmits over 100 plant viruses [2]. Its infestation causes massive agricultural losses every year [3–5]. Farmers use insecticides, including carbamates, organophosphates, pyrethroids and neonicotinoids to avoid yield losses.

Neonicotinoids, being nicotinic acetylcholine receptor (nAChRs) competitive modulators, effectively manage *M*. *persicae* [6]. Neonicotinoids captured a bulk of the annual pesticide sales after the introduction of imidacloprid in 1991 [7]. This overreliance and excessive use of neonicotinoids induced resistance in aphids [8]. The first report of neonicotinoid resistance in *M*. *persicae* dates back to 2007 in Greece. Moderate to high resistance against imidacloprid was observed in a few populations [9]. The field-evolved resistance to neonicotinoids in *M*. *persicae* has been reported from different countries [10–15].

Numerous factors contribute to evolution of resistance. Overexpression of cytochrome P450 monooxygenase and *E4/FE4-esterases* and mutation at *β1* subunit of nAChR cause varying levels of resistance to neonicotinoids [7]. The first study by Puinean et al. (2010) showed transcription level of a single P450 gene *CYP6CY3* enhanced to 22-fold of the control clone due to gene amplification in a resistant *M*. *persicae* clone (5191A) [16]. Similarly, an increased resistance level to imidacloprid in six Australian field populations of *M*. *persicae* showed a 2.8- to 6.7-fold increase in copy number of *CYP6CY3* [14]. An FRC *M*. *persicae* clone originated from southern France peach orchards presented resistance ratios up to 1679- and 225-fold to imidacloprid and thiamethoxam. The nAChR mutation (R81T) in the D loop region of β1 subunit was responsible for neonicotinoid resistance [17]. In 2012, a high-throughput assay was developed based on reverse-transcription polymerase chain reaction to study the spread and frequency of R81T mutation in *M*. *persicae* population originating from southern Europe. Results revealed high-frequency R81T mutation in field population collected from peach orchards in Gard, France. Subsequently, R81T mutation has been detected from several *M*. *persicae* populations, including Spain, Italy, Greece, and Tunisia, reflecting the range of an ongoing pest niche expansion around the Mediterranean basin [12, 15, 18].

Green peach aphid damages horticultural and field crops in China causing heavy economic losses every year. After the introduction of neonicotinoid insecticides in the early 2000s in China, these were extensively used to manage aphids and other pests. Several studies have addressed the development of multiple resistance levels to nicotinoids in the field population of *M*. *persicae* [4, 5]. Field population of aphids developed 19.42 and 1.95-fold resistance to imidacloprid and acetamiprid, respectively. Two field collected populations of aphids developing 6.03 to 6.51-fold resistance, and P450 cytochrome enzyme as key detoxifying enzyme conferring resistance against imidacloprid have been reported [4].

In the current study, first we investigated the resistance status of *M*. *persicae* to neonicotinoid insecticides and associated potential resistance mechanisms within field-collected population. Secondly, we validated the metabolic resistance mechanism targeting P450 *CYP6CY3* and *E4/FE4-esterases* genes using real-time quantitative PCR (RT-qPCR). Our findings provide timely information about the status and mechanisms of insecticide resistance in China, as well as recommendations for the management of *M*. *persicae* adaptive resistance.

## Materials and methods

### Ethics statement

No permission was required for insect collection, and species used is not regarded as endangered in the study area.

### *Myzus persicae* populations and rearing

*Myzus persicae* field population (FP) was collected from the Experimental Station of Lang fang, (GPS coordinates 116.6°E, 39.5°N), Chinese Academy of Agricultural Sciences (CAAS), Hebei, China during April 2017. Susceptible *M*. *persicae* clone (SC) was established from a population collected from the same site during 2013 and maintained in the laboratory with no insecticides exposure [19, 20]. Asexually reproduced aphids were fed on the leaves of Chinese cabbage (*Brassica napus* L. var *chinensis*) in rearing cages. Rearing conditions were 20–22°C temperature, 16h: 8h light-dark period and 65 ± 5% RH.

### Chemicals and reagents

Neonicotinoid insecticides, i.e., imidacloprid (analytical standard 96%), and acetamiprid (analytical standard 97.5%) were obtained from Shandong Lianhe Chemical Co., Ltd., China. Technical piperonyl butoxide, PBO (analytical grade 95%) was purchased from Shanghai Macklin Biochemical Co., China.

Takara DNA Marker DL1000 and Taq^TM^ DNA Polymerase were obtained from Clontech Takara, China. The TransScript^®^ One-Step gDNA Removal and cDNA synthesis SuperMix, 6×DNA loading buffer, TransStart^®^ Top Green qPCR SuperMix, nuclease-free water and GelStain (10000×) were all provided by TransGen Biotech Co., Ltd. RNeasy^®^ Mini Kit and QIAquick^®^ Gel Extraction Kit was obtained from Qiagen, ON, Canada. The rest of the chemicals and reagents used in the study were of analytical grade.

### Detection of insecticide resistance

The toxicity dose-response assay was performed according to leaf dip method as described previously [19]. Plastic discs were used to cut cabbage leaves, dipped in insecticide solution for few seconds (20–30 s), and air-dried at room temperature for 1–2 h. Thirty aphids of same age were inoculated onto the cabbage leaf surface placed in Petri dishes, 3 cm (Bio-Filtration Co., Ltd.) containing 1% agar solution. Petri dishes were sealed by Parafilm (Fisher Scientific, Ottawa, Canada) to prevent insect escape. Three replicates of each insecticide concentration were used, and the control group was only exposed to distilled water containing <1% EtOH. The bioassay response was assessed after 72 h. Aphids were scored as dead when slight or no movement was observed when probed with a fine brush. Probit analysis was conducted using SPSS statistical software (version 22.0) to calculate lethal median concentration LC_50_, slope, chi-square, and 95% confidence limits (CL). For each insecticide, the resistance factor (RF) was calculated as the LC_50_ value of the FP / LC_50_ value of SC.

### Synergist response assays

To determine the effect of cytochrome P450 enzymes, synergist PBO was used along with both insecticides in *M*. *persicae*. A screening diagnostic dose assay was performed to select sub-lethal doses of PBO for SC. Final concentration for PBO was 0.05 mg/L. The synergist factor (SF) was acquired by dividing the insecticide LC_50_ value alone by the LC_50_ value of the same insecticide synergized with PBO.

### Total RNA isolation and cDNA synthesis

A total of 15–20 aphids from FP and SC were used to pool as one biological replicate to extract RNA with Qiagen RNeasy^®^ mini-Kit (ON, Canada). The RNA quantification was calculated by the absorbance ratio at 260 and 280 nm using ND-1000 Nanodrop (NanoDrop Technologies, Wilmington, DE), and subjected to agarose gel electrophoresis for quality estimation. The cDNA synthesis was done through TransScript^®^ One-Step gDNA removal and cDNA Synthesis SuperMix (TransGen Biotech Co., Ltd, China). Three independent biological replicates were conducted for SC and FP.

### Quantitative real-time PCR

Expression profile observation of cytochrome P450 *CYP6CY3* gene was done using RT-qPCR. Moreover, PBO synergist shown inhibition of resistance-associated esterases [21]. The mRNA transcriptional levels of esterase *E4/EF4* were also detected in SC and FP to confirm the results of synergist bioassays. The primers to amplify 90–200 bp fragment of target genes and *β*-actin as an internal reference gene are listed in Table 1. The primers efficiency of each pair was assessed by 10-fold cDNA dilution. Twenty microliters of PCR reactions contained 0.4 μl each primer pair (10 μM), 10 μl 2×TransStart^®^ Top Green qPCR SuperMix, 1 μl template (cDNA), and variable ddH_2_O to make a total 20 μl volume. Samples were run on CFX Connect TM Real-Time System (BIO-RAD, Singapore). The thermal cyclic procedure contained an initial denaturation step at 94°C for 30 s, followed 40 cycles at 94°C for 30 s, 60°C for 30 s, and in last a dissociation step was executed to confirm the amplification of specified products. Each RT-qPCR experiment was included as independent three replicates. The RT-qPCR data for fold change of target genes was analyzed by the 2^-△△Ct^ method using the *β*-actin gene for normalization [22].

**Table 1:** Primers used in expression evaluation of cytochrome P450 *CYP6CY3* and esterase *E4* genes and sequence analysis of nAChR in *Myzus persicae*.

Genes	Primer Sequence (5´-3´)		Amplicon size (bp)	Reference
	Forward primer	Reverse primer		
R81T	GTCCAGAACATGACCGAAAAAG	CGCACAGGAAAGATATAAGGAC	619	[16]
CYP6CY3	CGGGGTGACGATCATCTATT	GGGTGGTCTTTTGACAAAGC	128	[16]
E4	AAACTTTCCTTTTACACCGTT	TCTAAGCCAAGAAATGTTGAAA	160	[16]
*β*-actin	GGTGTCTCACACACAGTGCC	CGGCGGTGGTGGTGAAGCTG	120	[16]

### Sequence analysis of nAChR

The presence and frequencies of mutation R81T in nAChR were analyzed using direct cDNA sequencing. Total RNA extracted from a single aphid was selected randomly from FP and SC with the acidic guanidine thiocyanate-phenol-chloroform method [23]. The RNA was subjected to 1.0% agarose gel to check quality. The cDNA was then synthesized using TransScript^®^ One-Step gDNA removal and cDNA Synthesis SuperMix (TransGen Biotech Co., Ltd, China). More than 50 individuals were used to extract RNA for each population to detect mutations in nAChR. Specific primers targeting a 619 bp fragment, including R81T mutation site in nAChR (accession# AJ251838) were chosen (Table 1) and synthesized by Beijing Genomics Institute. Cycling conditions for PCR were as follows: 95°C for 5 m, 95°C for 30 s, followed by 40 cycles of 56°C for 30 s, 72°C for 1 m, and a final extension at 72°C for 10 min. The PCR products were analyzed on 1% agarose gel, and amplicons were purified using QIAquick^®^ Gel Extraction Kit (Qiagen, ON, Canada). Purified products were sent to Beijing Genomics Institute for sequencing in both directions. The sequences of the required gene fragment were analyzed through DNAMAN 6.0 sequence analysis software. Three mutation genotypes were determined as susceptible homozygote (SS), resistant heterozygote (SR), and resistant homozygote (RR).

### Statistical analysis

One-way analysis of variance (ANOVA) followed by least significant difference (LSD) test was used to test significance in the data (transcriptional regulation) using SPSS software version 22.0. Results were considered significant when p value was <0.05. Median lethal concentration values (LC_50_) were determined through Probit analysis. Relative quantitative analysis (2^−ΔΔCt^) by Pfaffl, was used for calculating the fold change expression of targeted genes [21]. For the expression of relative quantities of *CYP6CY3* and *E4/FE4-esterases* genes, Tukey comparison was applied to test mean differences among FP and SC.

## Results

### *Myzus persicae* collected from Lang fang (FP) resistance to neonicotinoids

The LC_50_ values of the SC for imidacloprid and acetamiprid were 0.002 and 0.024 mg/L, respectively (Table 2). The LC_50_ value was 0.203 and 0.261 mg/L to imidacloprid and acetamiprid, respectively in FP. The *M*. *persicae* collected from Lang fang developed high-level resistance (101-fold) to imidacloprid and medium-level resistance (10.9-fold) to acetamiprid compared to SC.

**Table 2:** Dose-response toxicity bioassay of imidacloprid and acetamiprid to susceptible clone (SC) and field population (FP).

Population	Insecticide	LC_50_ (mg/L)	95%CL^a^	Slope (±SE)^b^	*df* ^c^	χ2^d^	*p*	RF^e^
			(mg/L)					
SC	Imidacloprid	0.002	0.001–0.003	0.89 (±0.15)	5	2.05	0.84	1.00
	Acetamiprid	0.024	0.017–0.034	1.41 (±0.18)	5	10.5	0.06	1.00
FP	Imidacloprid	0.203	0.084–0.845	1.04 (±0.16)	5	12.2	0.03	101
	Acetamiprid	0.261	0.177–0.389	1.13 (±0.17)	5	4.22	0.52	10.9

^*a*^Confidence limits;

^*b*^standard error;

^*c*^degrees of freedom;

^*d*^ Chi-square value;

^*e*^resistance factor

### Synergist bioassay of PBO in FP population compared to susceptible clone (SC)

The toxicity effect of PBO with insecticides was detected on *M*. *persicae* (Table 3). The PBO showed no synergism to imidacloprid and acetamiprid with the synergism factor of 1.00 and 0.96 in SC. In FP, synergism factor to imidacloprid and acetamiprid was 6.15 and 3.00, and the resistance level decreased from 101 and 10.9-fold to 16.5- and 3.48-fold, respectively. These results indicated that cytochrome P450 monooxygenase mediated resistance played a role in the resistance to neonicotinoids in FP.

**Table 3:** Synergistic effect of PBO on the toxicity of imidacloprid and acetamiprid to susceptible clone (SC) and field population (FP) of *M*. *persicae*.

Strain	Insecticide	LC_50_ (mg/L)	95%CL^a^	Slope (±SE)^b^	*df* ^c^	χ2^d^	*p*	RF^e^	SF^f^
			(mg/L)						
SC	Imidacloprid+PBO	0.002	0.002–0.004	0.974(±0.16)	5	2.73	0.74	1.00	1.00
	Acetamiprid+PBO	0.025	0.016–0.041	0.98 (±0.16)	5	2.55	0.77	1.00	0.96
FP	Imidacloprid+PBO	0.033	0.013–0.058	0.81 (±0.16)	5	2.50	0.78	16.5	6.15
	Acetamiprid+PBO	0.087	0.006–0.451	0.98 (±0.16)	5	20.1	0.01	3.48	3.00

^*a*^Confidence limits;

^*b*^standard error;

^*c*^degrees of freedom;

^*d*^Chi-square value;

^*e*^resistance factor;

^*f*^synergism factor

### Expression levels of cytochrome P450 *CYP6CY3* and esterase *E4/EF4* in SC clone and FP populations of *Myzus persicae*

The mRNA transcriptional levels of cytochrome P450 *CYP6CY3* were evaluated by RT-qPCR. The relative expression level of *CYP6CY3* gene in FP was 3.74-fold higher than SC (Fig 1A and 1B). The mRNA transcriptional levels of esterase *E4/EF4* were also evaluated with RT-qPCR to validate the result of synergic bioassay. The *E4/EF4* -esterase gene expression in FP was 1.51-fold of SC. Therefore, overproduction of *CYP6CY3* gene was associated with imidacloprid and acetamiprid resistance in field-collected *M*. *persicae*.

**Fig 1:** Relative mRNA transcriptional levels of (A) cytochrome P450 *CYP6CY3* and (B) *E4* in susceptible clone (SC) and field population (FP) of *Myzus persicae*. Data are presented as means ± SE from three independent experiments for each strain. The symbol (*) is used to denote significant difference (*p*<0.05).

### *Myzus persicae* sequence analysis of nAChR β1 subunit

Strong evidence of additional resistance mechanisms achieved in bioassays with a significant resistance factor remaining in FP to imidacloprid after PBO synergism. Therefore, the presence and frequencies of the R81T mutation in the loop D region of nAChR subunit *β1* in SC and FP were analyzed using direct cDNA sequencing (Table 4). A total 50 aphids of SC were observed in susceptible homozygous (SS). Among 50 aphids of FP, six were in homozygous resistant (RR), and fourteen aphids were present in the heterozygous form (SR). The resistance allele frequency (RAF) in FP was 26.0%. Additionally, two non-synonymous mutations at site Val^101^ (Val^101^Met, V^101^Ile) were detected in D loop region of nAChR subunit *β*1 of *M*. *persicae* (Fig 2). The RAF of V101M was 14%, while V101I displayed 32% frequency in FP. Interestingly, there were no other mutations when R81T mutation was present in homozygous form and there were no other mutations when V101I was present in homozygous form in nAChR. The schematic illustration of both mutations in *M*. *persicae* and their protein-coding sequences are presented in Fig 2. The potential role of mutations V101M (I) in the neonicotinoid resistance needs to be further studied.

**Fig 2:** Schematic of the *Myzus persicae* nicotinic acetylcholine receptor, the primary target of the neonicotinoids, showing a single mutation R81T position along with additionally found Val^101^Met, V^101^Ile mutations on *β*-subunit at loop D. Coding domain of loop D nAChR of R81 (45 bp) and V101 (110 bp) mutation is presented as A^G^A‒>A^C^A and ^G^TG‒>^A^TG / ^G^T^G^‒>^A^T^A^, respectively. Acetylcholine binding loop E and F are also presented on the protein-coding domain. Reproduced from [8, 24].

**Table 4:** Genotype and allelic frequencies of the R81T mutation in susceptible clone (SC) and field population (FP) of *Myzus persicae*.

Mutation	Population	*n* ^a^	Genotype			
			RR^b^	SR^c^	SS^d^	RAF (%)^e^
R81T	SC	50	0	0	50	0
	FP		6	14	30	26.0
V101M (I)	SC		0	0	50	0
	FP		2 (14)	10 (4)	20	14.0 (32.0)

^*a*^number of individuals;

^*b*^resistant homozygote;

^*c*^resistant heterozygote;

^*d*^susceptible homozygote;

^*e*^resistance allele frequency (RAF) = 100×(2×RR+SR)/2*n*.

## Discussion

Neonicotinoid insecticides are widely used to control *M*. *persicae* and rising concerns about decreased sensitivity necessitate monitoring of resistance and mechanisms against these compounds. Better management strategies are required to suppress or slow down the resistance phenomenon on urgent basis. The work described here focuses on *M*. *persicae*, a significant damaging crop insect pest to various hosts in China. Management of this pest is reliant on insecticides, including neonicotinoids. Recently, *M*. *persicae* has evolved resistance to neonicotinoids which are considered effective control in China [4, 5].

The insecticide resistance data showed that aphids collected from Lang fang station carried high (101-fold to imidacloprid) to moderate (10.9-fold to acetamiprid) levels of resistance against two neonicotinoids compared to a susceptible clone (SC). Cases of reduced susceptibility to neonicotinoids in *M*. *persicae* has been described in several field populations collected from different sites of China. Tang et al. [5] reported Lang fang field population collected in 2013 developed 19.42- and 1.95-fold resistance to imidacloprid and acetamiprid, respectively. It shows an obvious variation in the level of resistance to imidacloprid and acetamiprid, which could indicate a potential for the development of resistance.

Cytochrome P450 encoding gene *CYP6CY3* overexpression has been linked with neonicotinoids resistance in *M*. *persicae* field populations globally [14]. In the present study, resistance of neonicotinoids was associated with enhanced detoxification by cytochrome P450 enzymes in FP, which was documented initially by results of synergist PBO bioassays. In FP, the synergism factor of PBO to imidacloprid and acetamiprid was 6.15 and 3.00, and the resistance level decreased from 101- and 10.9-fold to 16.5- and 3.48-fold, respectively. The mRNA transcriptional level of *CYP6CY3* gene was significantly (*p*<0.05) increased in FP compared to SC. In our previous study, FP was exposed to sub-lethal toxicities of acetamiprid and imidacloprid over consecutive 04 generations and then expression of P450 cytochrome gene *CYP6CY3* was enhanced to 5.47- and 5.20-fold [19]. These results confirmed that the increased level of mRNA transcription of gene *CYP6CY3* was associated with neonicotinoids in *M*. *persicae*.

Concerning the neonicotinoids target-site resistance in *M*. *persicae*, R81T mutation at nAChR *β1* subunit was first detected in France. In 2012, Puinean et al. [24] detected the R81T substitution by developing a real-time TaqMan assay and to observe the frequency of the R81T mutation in collected aphids and stored in ethanol from peach orchards in southern France. The R81T mutation frequency varied from 33 to 100% in 7 populations. Similarly, R81T mutation was present at large frequencies (32–55%) in aphids collected between 2014 and 2016 in Tunisia [15]. In this study, detection of single point R81T mutation was observed in *M*. *persicae* FP collected from Lang fang City, China. The resistance allele frequency (RAF) in FP was 26.0% (12.0% for homozygous allele and 14.0% for heterozygous allele), which showed 101-fold to imidacloprid and 10.9-fold to acetamiprid compared to SC. Mottet et al. [25] assessed dominance status of R81T mutation to imidacloprid and thiacloprid in 23 *M*. *persicae* clones *in vitro*. Their results showed all homozygous genotypes of clones for R81T substitution and indicated maximum resistance to both tested neonicotinoids than wild and heterozygous clones. The heterozygous clones exhibited a little higher resistance level than homozygous wild. Moreover, mutation R81T conferred greater resistance level to nitro-substituted neonicotinoid, such as imidacloprid, than to cyano-substituted neonicotinoid, such as acetamiprid [26]. This information corroborated our results that FP showed 101-fold resistance to imidacloprid, but only 10.9-fold resistance to acetamiprid. Another two non-synonymous mutations Val^**101**^Met and V^**101**^Ile, were also found in the conserved domain of nAChR subunit *β*1; however, their role in the neonicotinoid resistance warrants further investigation. Anyhow, the present research gives useful information for resistance monitoring and will aid in the development of *M*. *persicae* adaptive resistance management tactics in China.

## Conclusion

The collected aphids from Lang fang station carried a high to moderate resistance level to both neonicotinoids. Cytochrome P450 enzyme and R81T mutation in nAChR were involved in developing neonicotinoid resistance. Two other non-synonymous mutations Val^101^Met and V^101^Ile were also found in nAChR subunit *β*1, and their potential role in resistance warrants further investigation. Our results offered a basis for ascertaining sustained *M*. *persicae* susceptibility to neonicotinoid insecticides and conserving the field efficacy of this class of insecticides.

## Supporting information

S1 Data (XLSX)
